# A Multimodal Convolutional Neural Network Model for the Analysis of Music Genre on Children's Emotions Influence Intelligence

**DOI:** 10.1155/2022/5611456

**Published:** 2022-08-29

**Authors:** Wei Chen, Guobin Wu

**Affiliations:** Changchun Humanities and Sciences College, Changchun 130117, Jilin, China

## Abstract

This paper designs a multimodal convolutional neural network model for the intelligent analysis of the influence of music genres on children's emotions by constructing a multimodal convolutional neural network model and profoundly analyzing the impact of music genres on children's feelings. Considering the diversity of music genre features in the audio power spectrogram, the Mel filtering method is used in the feature extraction stage to ensure the effective retention of the genre feature attributes of the audio signal by dimensional reduction of the Mel filtered signal, deepening the differences of the extracted features between different genres, and to reduce the input size and expand the model training scale in the model input stage, the audio power spectrogram obtained by feature extraction is cut the MSCN-LSTM consists of two modules: multiscale convolutional kernel convolutional neural network and long and short term memory network. The MSCNN network is used to extract the EEG signal features, the LSTM network is used to remove the temporal characteristics of the eye-movement signal, and the feature fusion is done by feature-level fusion. The multimodal signal has a higher emotion classification accuracy than the unimodal signal, and the average accuracy of emotion quadruple classification based on a 6-channel EEG signal, and children's multimodal signal reaches 97.94%. After pretraining with the MSD (Million Song Dataset) dataset in this paper, the model effect was further improved significantly. The accuracy of the Dense Inception network improved to 91.0% and 89.91% on the GTZAN dataset and ISMIR2004 dataset, respectively, proving that the Dense Inception network's effectiveness and advancedness of the Dense Inception network were demonstrated.

## 1. Introduction

Emotions are fundamental to our daily lives and play an essential role in rational decision-making, perception, healthcare, and human intelligence [1]. However, affective states are primarily overlooked, so the use of computers to analyze and process affective signals from sensors to identify a person's affective state has become a hot topic of contemporary research. There is no strict range calibration to differentiate musical works of different genres in terms of rhythmic and genre-specific expression features. However, other musical results of the same genre express their properties similarly. By capturing the similarity patterns unique to the same genre, it is possible to determine the genre attributes in musical expression. Such similarity patterns are universally applicable, allowing classification operations with more significant data sizes to be accomplished [2]. Traditional music genre classification methods are mainly achieved through manual or social annotation. Manual classification requires participants to have a certain degree of music expertise. Although it can ensure the classification effect, manual sort consumes much labor and time and is also costly. Although this classification mode saves costs, it is not easy to guarantee its classification effect [3].

One of the critical aspects of multimodal sentiment recognition is the fusion strategy. In machine learning, multimodal fusion usually employs feature, decision, and hybrid fusion [4]. Although these methods can perform well in multimodal sentiment recognition, they are shallow fusion models that perform poorly in uniting and modeling multiple input features. Some new approaches have been recently investigated in the field of emotion recognition, which fuses the information of all available modalities directly with deep learning networks for feature extraction and optimization, which can achieve the fusion of multiple modalities into a single modality to enhance the stability of the recognition process [5]. A profound sentiment recognition model based on multimodal decomposition bilinear pooling is proposed. In this model, we first select the channels of EEG signals to reduce the interference caused by redundant channels. Then, convolutional neural networks extract each modality's convolutional features [6]. Finally, a multimodal decomposition bilinear pooling method is used to fuse and optimize the characteristics of each modality. The proposed fusion strategy allows all elements of each modality to interact to express each modality's complex internal relationships effectively. The model has an average accuracy of 93.22% on the DEAP dataset and 90.50% on the MAHNOB-HCI dataset, demonstrating that the model can improve multimodal sentiment recognition performance and significantly outperform existing techniques.

Neural networks have led the development of artificial intelligence in recent years, among which Convolutional Neural Networks (CNN) is a leader in image recognition, which can find out the features in complex images with high accuracy, improvement space, and sound processing efficiency in the face of high-dimensional data, and its architecture and each component element are still developing rapidly. On the other hand, there are many good deep algorithms available. On the other hand, many excellent deep learning frameworks are no longer challenging to build an easy-to-use deep learning system [7]. The development of computer hardware also gradually decreases the computational cost, making deep learning algorithm models such as convolutional neural networks closer to daily life [8]. This paper uses music genre classification and recognition as the research direction; we use short-time Fourier transform, Meier transforms, and constant *Q* transform to process one-dimensional audio files to generate spectrum and related data and use a convolutional neural network to automatically learn to extract acoustic features such as rhythm, pitch, and chord from images to build a music genre classification model. Applying deep learning techniques combined with EEG signals for multimodal emotion recognition methods has become a research trend [9]. This paper addresses the issues related to feature extraction and feature fusion in multimodal emotion recognition: on the one hand, we propose a layered fusion feature extraction to improve the recognition rate of emotion states; on the other hand, we use deep learning models to automatically extract and fuse multimodal signal features based on bilinear pooling of multimodal decomposition to achieve intelligent analysis of the influence of music genres on children's emotions.

## 2. Related Works

With its unique artistic elements of melody, rhythm, and harmony, music is significantly more complex than ordinary audio in terms of sound composition. The different ways of combining other artistic elements in a musical work while designing various musical works also produces different genres to which the musical works belong [10]. When enjoying a musical work, in addition to the singer's voice and the performer's song, there will be the presence of other combinations of elements such as natural sounds and frequencies outside the range of the human ear's vocal range. In the early days, when musical genre classification arose, humans could determine the genre affiliation of different music by analyzing it. However, the way humans understand and perceive music is challenging to construct through scientific methods, so it is not easy to implement automated music genre classification to allow computers to process it according to human determinations [11]. Since the introduction of automatic genre classification, extracting music's audio signal and processing it by machine learning models can effectively realize the automatic determination of music genre attribution [12]. The research on music genre classification has continued to focus on the extraction of features expressing musical attributes and attribute decisions based on the extracted features, among which the extraction of features describing musical details is the most significant [13]. In music genre classification, the study of feature engineering has been proposed since the 1990s. Gu et al. analyzed and verified the effectiveness of genre classification models based on sparse representation by introducing audio features such as spectral variance and combining them with principal component analysis methods for data dimensionality reduction [14]. Li et al. analyzed the GTZAN dataset and found some problems through targeted experimental design, which provided the relevant basis for the subsequent academic work of researchers [15].

Compared with unimodal sentiment analysis, multimodal sentiment analysis can overcome the noise effect carried by unimodal modality on the one hand and retain the practical information of each modality based on the complementary characteristics of different modalities on the other hand. Pan et al. combined LSTM and attention mechanism to extract the emotional relationship between contextual discourse in the video and introduced multimodal context-dependent information further to improve multimodal sentiment analysis systems [16]. Although all the research works in recent years have advanced the development of multimodal sentiment analysis to some extent, there are still problems such as limited characterization ability of unimodal sentiment features, insufficient robustness of fusion models, and no characterization ability of fused multimodal sentiment features. Based on the previous work, there is a need and feasibility to continue in-depth research [17]. Perceptual inconsistencies make it insufficient to predict highly personal variables' central (average) effective category [18]. Gonzalez et al. propose that two multimodal affective computing tasks can be performed to deal with the subjectivity challenge: predicting each viewer's individualized affective perception and assigning multiple influential labels to each stimulus [19].

The child's inner emotional power system is the pillar of a balanced education. Moral, intellectual, emotional, aesthetic, creative, and physical elements constitute the spiritual world of each child [20]. When influencing children, it is necessary to educate them not only about knowledge but also about the development of their personality. Therefore, the product of emotions is an essential guarantee for the child's comprehensive development [21]. To improve the one-sidedness and deformation of educational development, we must pay attention to the role of emotions in the educational process. He believes that the key to the stimulation of children's “emotional motivation” lies in the teacher, who should have the art of mastering children's thinking, be highly perceptive and flexible, change teaching methods at any time, be good at encouraging children in teaching activities, care about children's life and health, their interests and happiness, and their complete spiritual life. Teachers and students should make spiritual contact, stimulate children's sense of self-esteem, self-confidence, and trust in teachers and make children enjoy learning success.

## 3. Multimodal Convolutional Neural Network Model Construction

Convolutional neural networks (CNNs) are now a common type of feedforward neural network and have an important position in the field of computer vision; the convolutional effect of CNNs can handle the correlation information in adjacent local receptive fields, and in computer vision problems, CNNs do not need to use one-to-one connections between all pixel units (i.e., like most neural networks), but instead use grouped local links. In addition, another feature of CNNs is the shared weights, where the convolutional kernel uses the same importance at all positions in the same layer, so the size of the network parameters can be effectively reduced [22]. As the depth of the network increases, the increase in the size of the sensory domain allows the network to represent more abstract features of the input. The convolutional layers focus on the edge portion of the object and then process the entire thing at a higher level in the hierarchy. Gradient descent combined with error backpropagation is essential for solving multilayer networks. A convolutional neural network is a multilayer structure that contains a feature extractor consisting of several convolutional layers, subsampling layers, and a connection layer. A neuron is connected to only some of its neighboring neurons in a convolutional layer. A convolutional layer in a CNN usually contains several feature maps, each consisting of several rectangularly arranged neurons that share the weights of the same feature map. The shared consequences are the convolution kernels. The convolution kernel is usually initialized in the form of a random fractional matrix, and the seed will learn reasonable weights during the training process of the network.

(1) $$\begin{array}{c} w_{\left(k-1\right)}=\sum \frac{\sqrt{\partial e\left(w-1\right)+\alpha }}{\sqrt{w_{k-1}-\partial w}}. \end{array}$$

The gradient is calculated on the training set. The gradient descent equation can be easily solved using the chain rule of derivatives. An image input of 25 ∗ 25 pixels in size is an example of handwritten digit recognition. The information in the convolutional network is arranged as an array of 25 ∗ 25 design warp elements arranged in a rectangle, and their values correspond to the 25 ∗ 25 pixels used as the input. By convention, the input pixels are connected to the implicit layer neurons. However, CNN differs from fully connected layers in that CNN establishes connections.

(2) $$\begin{array}{c} \sigma =\sum \frac{w_{1}-m_{a}-a_{x,y}}{\sqrt{b-l-m}}+\sqrt{k-m}, \end{array}$$

where *σ* is the activation function of the neuron, possibly a sigmoid function, *b* is the shared bias, *w*_1,*m*_ is the 5 ∗ 5 shared weight matrix. *a*_*x*,*y*_ denotes the input excitation at positions *xy*. All neurons in the first hidden layer detect a particular feature at a different location in the input image. To justify this setup, assume that a certain weight and bias, i.e., a hidden neuron, can detect vertical edges. This ability may also be functional elsewhere in the image. Thus, the same feature detector can be applied anywhere in the picture. To perform image recognition, we need multiple feature mappings, and one convolutional layer corresponds to many different feature mappings, as shown in Figure 1.

This structural design detects many different features and can be performed from any position in the graph. One outstanding advantage of shared importance and tendencies in convolutional neural networks over fully connected neural networks is that it dramatically reduces the size of the network parameters. If every input pixel were fully connected to a neuron in the hidden layer, it would require roughly 40 times more parameters in this example. The training process of deep convolutional neural networks can also converge quickly. The mathematical equation describes the process of moving neurons from input to output.

(3) $$\begin{array}{c} y=\sum_{i=1}\left(n-x_{i}\right)\times w_{i+b}+\sqrt{f-1}. \end{array}$$

A neuron's input can come from the input signal and the output of other neurons. This fully connected neural network has many neurons, divided into three layers, from top to bottom. The network structure has only one hidden layer; this neural network is called single hidden layer feedforward neural network. In deep learning, multiple hidden layers can be set up, and each hidden layer has a different number of neurons according to the actual situation to improve the learning ability.

For the hidden and output layers, the connection weight matrix of each layer with the previous layer and the output value of the neurons in the last layer are multiplied by the bias term of that layer to obtain the linear output [23]. Then the activation function of that layer is nonlinearly transformed to get the work of the neurons in that layer. The computational equation describes the process of the neuron in each layer, from receiving the input to computing the output.

(4) $$\begin{array}{c} z^{l}=\int_{l=1}\frac{b^{L}-1}{w^{L}+a^{L+1}}, \end{array}$$

(5) $$\begin{array}{c} a^{l}=\sum \frac{f^{L}+z^{L}}{\sqrt{f^{L}-z^{L}}}. \end{array}$$

Equation (4) is the linear output vector of the neuron at the first layer, calculated from the output vector of the neuron at the coating *L* − 1*a*^*L*−1^, the connection weight matrix at the layer *LW*^*L*^ , and the bias term at the *L* layer *b*^*L*^. In equation (5), *a*^*L*^ is the nonlinear output vector of the neuron at layer *L* obtained by passing the linear output of the neuron at layer *Lz*^*L*^ through the activation function *Lf*^*L*^(*·*). Starting from the input layer, along with the input to output direction, as in the above process, the input vector, connected weight matrix, and bias term of each layer are subjected to a series of linear and activation operations and computed layer by layer backward until the target prediction result is obtained in the output layer, such a process is the forward propagation process. An LSTM network contains three gates: forget, input, and output. The forget gate is used to remove redundant information, while the input gate is responsible for updating the old cell state, and the output gate affects which part of the output of the updated cell state. Advantageous in sequence modeling problems with long-time memory. Simple to implement. Solve the problem of gradient disappearance and gradient explosion in the long sequence training process.

(6) $$\begin{array}{c} Z=\sum \tanh\frac{1-b}{\sqrt{\theta x^{T}-zwh^{T-1}-B}},\\ z-l=\sum \tanh\frac{zwh^{T-1}}{\theta x^{T}-zwh^{T-1}+B},\\ z^{f}=\sum \frac{Bf-1}{\sqrt{\theta_{f}x^{T}-W_{f}h^{T-1}+Bf}}. \end{array}$$

## 4. Design of an Intelligent Analysis Model of the Influence of Music Genres on Children's Emotions

The most significant difficulty in feature selection for music classification can be solved by deep learning models, which allow computers to automatically learn the pattern features needed to correctly classify music, making it possible to design effective models without relying on a deep knowledge of audio signal processing and music theory. Many studies follow image processing experience in designing convolutional neural networks, lacking an effective method for feature attributes in music audio spectrograms [24]. In this section, this paper proposes a residual module and a dual-attention fusion module for music feature extraction that combines residual the model in extracting high-dimensional abstract features of music by stacking residual modules and enhancing the directionality of feature extraction by dual-attention fusion modules, thus optimizing the training efficiency of the model and thus improving the effectiveness of music genre classification.

The DCNN-AFC model performs Mayer filtering on the original audio signal, converts the filtered audio signal into an audio spectrogram, and then splits it into DCNN. Model training, the model, completes the training and validation of the corresponding music data on the training and validation sets as a batch for multiple iterations and outputs the model when it reaches the specified collection. The DCNN-AFC model flow is shown in Figure 2.

Given the ability of DCNN to extract features in the audio spectrogram and the performance of audio spectrogram classification, the residual structure, channel attention mechanism, and spatial attention mechanism are introduced to enhance the model's performance in extracting audio spectrogram features. The partial design of the network is improved to propose a deep convolutional neural network model consisting of an effective combination of the residual module, and dual-attention fusion module.

Six features are selected: chromatic frequency, root mean square of the spectrum, the spectral center of mass, acoustic spectrum roll-off coefficient, Mel frequency cepstral coefficient, and over-zero rate. Their mean values are calculated, and the mean values of 20 features of the Mel frequency cepstral coefficient are added to form a total combination of twenty-six features to describe the feature information of a piece of music. And the classification model is designed as a hybrid model containing an LSTM submodule and one-dimensional convolutional submodule according to the characteristics of feature combination, and the performance of traditional LSTM and LSTM containing attention mechanism in the model is compared. Through continuous exploration of acoustics, we have extracted acoustic features from various aspects, and digitized music can often remove hundreds of dimensional acoustic features. The audio spectrum of an audio signal is shown in Figure 3.

Music teaching is not only for all children but should also be able to take special care of and accommodate children. This is not for music teachers to treat children differently, but to teach in detail so that children no longer feel alone but love and care from the inside, making them feel happy and successful in learning music. The content of music teaching should be appropriately integrated with children's lives, able to express children's hearts, pay attention to children's interests, attitudes and needs, strengthen the emotional experience, improve children's ability to externalize their emotions, and make children more adept at using music to regulate and express their feelings. Music teaching should be carried out in a relaxed, friendly, and pleasant environment, focusing on nurturing; the teaching language should be mainly encouraging, providing children with rich ways of participating in musical activities and opportunities for expression, cultivating their cheerful character, enhancing children's self-confidence, cultivating their strong will and courage to face, and overcome difficulties, and developing their optimistic attitude toward life and living. To realize big comprehensive data intelligent analysis, this section examines establishing a cross-platform unified big data programming model covering the table, matrix, tensor, graph, and streaming data models. It then further explores the construction of a programming method for big data intelligent analysis based on computational flow graphs. The big data brilliant analysis programming model and framework are shown in Figure 4.

At the same time, the upper-layer analytic algorithms and applications are implemented based on platform-independent high-level programming computational models and interfaces [25]. Through the cross-platform unified high-level abstract big data programming computing model and interface, the upper-layer data analysis algorithms and applications can be decoupled from the underlying distributed parallel computing platform, hiding the details of the underlying big data computing platform from the upper-layer data analysts, realizing the transparency of the underlying platform to the upper-layer algorithm design and application development, and thus significantly improving the ease of use of the big data processing system platform.

## 5. Analysis of Results

### 5.1. Analysis of Multimodal Convolutional Neural Network Models

To verify the effectiveness of the multimodal convolutional neural network proposed in this chapter, 62 channels of EEG data and eye-movement data of the subject children in the SEED-IV dataset were used as experimental data. In the unimodal signal-based emotion recognition experiments, the MSCNN network was used to classify the 62-channel EEG data for emotion. Single-modality image alignment refers to the floating two images acquired with the same imaging device. It is mainly applied to the alignment between different MRI-weighted images and the alignment of image sequences, etc. Multimodal image alignment refers to the floating of two images from other imaging devices. The LSTM network was used to realize the emotion classification based on the eye-movement signal; the MSCNN-LSTM model was used for the multimodal signal emotion classification experiments. Three experimental data for each child at different periods were conducted separately, with a total of 45 experiments. Each sample size of EEG data was 5 × 62, each sample size of eye-movement data was 1 × 31, and the total sample size of session 3 was 812. First, the samples were preprocessed. After normalization with zero-mean normalization, the training set and test set are divided according to the ratio of 8 : 2, and the number of experimental iterations is set to 300. In terms of emotion classification, the eye-movement signal contains less obvious emotion recognition features than the EEG signal and multimodal signal, and the EEG signal and multimodal signal are more suitable as data for emotion classification studies; second, the experimental results of different signals all that the accuracy rates of the first experiment and the second experiment are generally higher than those of the third experiment, which may be due to the acquisition environment of the third experiment or other factors may have influenced the data acquisition in the third experiment. The comparison of the classification results of unimodal and multimodal signals is shown in Figure 5.

The advantages of multimodal signals relative more intuitively to unimodal signals, the average accuracy of subjects' emotion classification in three experiments under three different signals and the average classification accuracy in 45 experiments under three separate signals, where the three different signals were 62-channel EEG signal, eye-movement signal and 62-channel EEG signal fused with eye-movement signal in the multimodal signal. From the experimental results, in the first eight subjects and the last two subjects, the classification accuracy of the emotion of multimodal signal is higher than that of the unimodal signal. In contrast, the classification results of subject 9, subject 10, subject 11, subject 12, and subject 13 showed that the classification accuracy of the emotion of multimodal signal is lower than that of unimodal signal, which means that multimodal convolutional neural network has subject variability from the side; the classification accuracy based on the multimodal signal. The average accuracy of 45 experiments based on multimodal signals, EEG signals, and eye-movement signals are 95.2139%, 96.2315%, and 93.0641%, respectively. However, multimodal signals have individual differences; for most subjects, the accuracy of multimodal-based emotion classification is higher than that of unimodal signals, which verifies the effectiveness of multimodal signals and verifies the efficacy of multimodal convolutional neural networks for emotion classification of multimodal signals.

When the parameters in the DEAP dataset were optimal, the average accuracy of the wakeup dimension was 83.28%, and the valence dimension was 84.71%. When the parameters in the MAHNOB-HCI dataset are optimal, the accuracy of the wake dimension is 88.28%, and the valence dimension is 89.00%. It can be concluded that the model performs better in the valence dimension than in the wake dimension using the same dataset with optimized parameters, which indicates that the model proposed in this chapter is more active in the valence dimension [26]. When the classifier parameters are optimal, the accuracy of the model presented in this chapter applied to the MAHNOB-HCI dataset is higher than that of the model applied to the DEAP dataset. The experimental results obtained using a layered fusion convolutional neural network to extract features are significantly better than those obtained using only the convolutional neural network alone. The reason is that although convolutional neural networks can automatically learn and extract multilayer feature representations from the original data, the neural network does not focus on one feature per neuron; instead, a group of neurons focuses on one part. The variation curves of classifier accuracy with parameter settings are shown in Figure 6.

### 5.2. Intelligent Analysis of the Impact of Music Genres on Children's Emotions Realized

The music genre includes many sensory systems, such as visual, auditory, and tactile. The first sense that needs to be used is visible, which transmits the notes on the music score to the brain's nervous system. This is followed by the sense of hearing, which is the inner sense of hearing, a mental activity based on the perception of music and the purpose of shaping musical images; that is to say, the inner meaning of hearing at this time is a kind of auditory imagination of the expected music and the effect of the music style. Next, the natural sound is put out through kinesthetic and tactile senses, and only then does the honest auditory feedback appear. Therefore, the coordination of the sensory and motor systems is the most critical psychological basis for improving the coordination of musical movements. First, sight-reading skills can be enhanced through sight-singing and ear-training exercises, which allow children to connect music and sound and vision and hearing. Second, children can perform the sighted scores so that they can establish connections between the scores and performance, visual and kinesthetic senses, and strengthen their inner auditory and tactile senses so that the sensory system and the motor system will gradually coordinate, and the coordination of movements in music performance will improve progressively. Of course, it is also possible to use the Dalcroze somatic rhythm teaching method to enhance the connection between children's auditory and kinesthetic senses so that children can feel the relationship between music and movement and improve the coordination between hearing and kinesthetic senses. To illustrate the effect of the number of iterations on model training, experiments were conducted on the validation set with a learning rate of 0.01 and 37,000 iterations. The genre classification accuracy plot for 37000 iterations is shown in Figure 7.

The audio fragment-based prediction method can make the model more flexible to cope with different time-length music samples, which is very important in practical use. According to the previous settings, 66560 sampling points at 22050 Hz audio are used as an audio clip. The audio clips are selected by randomly selecting the starting point and sequentially intercepting the audio clips. There is a 50% overlap between the audio clips, which avoids the loss of information partially located near the audio clip interception point across the two audio clips due to nonoverlapping cutting. The model's performance was tested in the prediction phase using different numbers of segments from 1 to 18, and the classification accuracy in the prediction phase using other numbers of features is shown in Figure 8. The accuracy of the model increases rapidly as the number of audio segments increases when the model uses a small number of pieces for prediction; from using one audio component for prediction to using ten audio details for prediction, the accuracy improves by about 3.87% after smoothing (the accuracy improves by about 5.1% before filing). As the number of audio clips increases, the model's accuracy increases slower, from using ten audio clips for prediction to 18 audio clips, with an improvement of about 8% after smoothing (and about 0.4% before filing). Theoretically, increasing the number of audio clips used for the prediction can improve accuracy. Still, as the number of audio clips used increases, each audio clip will bring less and less additional valid information and will contribute less and less to the accuracy improvement. Eventually, the accuracy will converge to a stable interval, so it is not meant to increase the number of audio clips used blindly. To ensure a high accuracy rate while avoiding a meaningless increase in the number of audio clips and combining the characteristics of the GTZAN dataset, 18 is finally chosen as the number of audio clips used in the prediction stage of the model.

The intelligent analysis dataset was divided into equal proportions according to the category labels with the ratio of 80%, 10%, and 10% for the training set, validation set, and test set, respectively. In total, 200 rounds were conducted on the training set using a learning rate of 0.001, and the learning process was supervised using the validation set. The training was terminated early when the accuracy performance on the validation set did not improve for more than 20 rounds. A total of about 219 hours of training was conducted, and the activity was terminated early after 8 games of movement without any further improvement in accuracy on the validation set. The pretrained model was used as the base model for migration learning. The last fully connected layer was replaced according to the number of categories in the GTZAN, ISMIR2004 dataset, and retrained as a starting point. After the same training process with the exact details described in the previous section, the model classification accuracy was improved substantially. The model's 10-fold cross-validation classification accuracy was improved to 91.0% and 89.91% on the GTZAN and ISMIR2004 datasets, respectively, as shown in Figure 9. Music genres begin with auditory sensations and express auditory content by triggering emotions through auditory senses. Thus, music genres strengthen the connection between aural and kinesthetic feelings and music and emotions. It is believed that the problem of children's coordination of movements in musical genres is caused by the lack of close coordination between the neurological system of the child's brain and the parts of the body and the separation of the child's mind and body from the music felt in musical genres. In music genres, children can feel the fusion of emotions and music, experience muscle tension and relaxation, strengthen the connection between the brain's nervous system and body parts, and improve the coordination of body parts, which are precisely the causes of children's emotions. Therefore, it is believed that the use of the music genre has a vital role in promoting the coordination of movements in the emotional impact of children.

## 6. Conclusion

As a critical technology in the development of computer intelligence, emotion recognition has significant application research value for guiding machines to serve human beings better. However, because human emotions are complex and diverse, it is challenging to accurately grasp specific emotional attributes and categories. Numerous challenges in this field still need to be tackled and solved by researchers. In this paper, we design a deep convolutional neural network-based music genre classification (DCNN-AFC) model to determine the genre attributes of musical works by processing the audio spectrogram of audio signals through dimensionality-reduced Mel filtering and capturing the gene expression features of music files. In this paper, a sub-dataset generated from the MSD dataset is used to pretrain the Dense Inception network, and then the pretrained model is used to train on the GTZAN dataset and the ISMIR2004 dataset. This pretraining step improves the stability of the model and the convergence during training while significantly improving the classification accuracy of multiple datasets. Comparing before and after pretraining using the MSD dataset, the accuracy of the Dense Inception network improved from 88.7% and 87.68% to 91.0% and 89.91% on the GTZAN dataset and the ISMIR2004 dataset, respectively. The use of computer-based interactive teaching not only updates the traditional teaching methods and enriches the teaching contents but also makes the abstract music realistic and lively, which significantly broadens children's musical horizons, enlivens their musical thinking, stimulates their enthusiasm for learning music, and increases the efficiency of analyzing children's emotional impact. Although the multimodal emotion recognition system designed and developed in this paper functionally realizes the recognition and visualization of students' learning emotions, the form of visualization presentation is relatively single, and consideration can be given to increasing the diversity of visualization presentation content. Since the system is operated based on separate computer local storage, the management of student data and course data is cumbersome, after which the use of a database for user data and course data should be considered. Control, to simplify the operation of users, while the effect of providing feedback to teacher users should be analyzed and designed according to the actual user needs, and more feasible functions should be added based on giving visual input to improve the practicality of the system.

## Figures and Tables

**Figure 1:** Convolutional layers corresponding to different feature mappings.

**Figure 2:** DCNN-AFC model flow.

**Figure 3:** Audio spectrum of the audio signal.

**Figure 4:** Data intelligence analytics programming model and programming framework.

**Figure 5:** Comparison of classification results between unimodal and multimodal signals.

**Figure 6:** Variation curve of classifier accuracy with parameter settings.

**Figure 7:** 37000 iterations of genre classification accuracy graph.

**Figure 8:** Classification accuracy when using a different number of segments in the prediction stage.

**Figure 9:** Accuracy comparison before and after using intelligent analysis dataset.

## Data Availability

The data used to support the findings of this study are available from the corresponding author upon request.
